# Research on the Driving Factors of Constructing Innovative Thinking Environment from the Perspective of Online Community

**DOI:** 10.1155/2022/6063418

**Published:** 2022-07-05

**Authors:** Xin Xin, Wanqing Shi

**Affiliations:** ^1^Jilin University, School of Philosophy and Society, Changchun 130012, Jilin, China; ^2^Jilin International Studies University, School of Marxism, Changchun 130012, Jilin, China

## Abstract

With the development of Internet information technology, the Internet space and the real space are increasingly integrated, and the influence of the Internet community has surpassed the cyberspace. The online community is not only a product of virtual space, but also integrates with the real society in terms of community interaction mode, network communityization of geographic communities, and dematerialization of social organizations. This offline integration trend objectively requires changes in online community governance at the level of thinking and system. Internet governance and social governance should be integrated to build a diversified, collaborative, and intelligent innovative online social governance system. This paper discusses the factors of creative thinking from the perspective of online community. Therefore, from the perspective of online community, more attention should be paid to the innovative thinking of online community, and the online community itself should play a more important role in the online social governance system.

## 1. Introduction

Network community generally refers to the human social group formed on the Internet. Different from social groups and organizations in the traditional sense, the formation, activities, and evolution of online communities were initially carried out in the Internet space. In the view of early researchers, online community has a kind of virtual reality, and many scholars focus on the virtuality and other characteristics of online community.

However, with the wide application of the Internet in economic, political, and social life around the world, the Internet space and social space in the traditional sense are being merged in a realistic sense [1]. On the one hand, more and more real social life takes place on the Internet, and social actions that originally needed to take place in the physical scene can be realized in the Internet scene [2]. On the other hand, network actions that originally only occurred in the Internet scene have an increasingly important real-world social impact and in some cases are directly related to real public issues and the relationship between the people and the state [3]. Therefore, in the network social governance system, the governance of the network community should be paid more attention, and the network community itself should also play a more important role in the network society governance system.

With the advent of the Internet information age, research-based learning based on the Internet has radiated new vitality [4]. The Internet is rich in information resources, an open environment, smooth interaction, convenient data collection, and easy-to-use information tools (Figure 1), which provides a reliable guarantee for the construction of educational informatization and the implementation of research-based learning in colleges and universities, which is not only conducive to teachers and students to carry out research-based learning, but also conducive to the cultivation of students' creative thinking ability [5].

Today, with the increasing development of science and technology, we clearly see that cultivating innovative talents is the call of the times, and the most important thing in cultivating innovative talents is how to cultivate their creative thinking [6]. Creative thinking has the characteristics of randomness, flexibility, uniqueness, and uniqueness, so it puts forward higher requirements for the cultivation of new talents, not only with keen observation, rich imagination, but also with new things. Prediction and evaluation abilities are developing rapidly, and Internet network teaching just meets the requirements of cultivating these abilities and qualities.

## 2. A Review of Related Research at Home and Abroad

In 1993, the concept of “Network Community” was first proposed by Howard Rheingold as “Virtual Community,” which has caused widespread concern in psychology, behavior, and informatics. Scholars in sociology, library science, media science, economics, and other fields have different concerns [7]. Foreign research on online communities has strong academic rationality and regards online communities as a form of social connection for real people to gather in the Internet field [8]. Quentin Jones believes that the composition of online communities needs to meet at least four conditions: the ability to interact, different types of communicator, the presence of enduring members, and a virtual public space that hosts interactions [9]. Domestic scholars believe that understanding the differences between online communities and real communities can be an important perspective for defining online communities, and they believe that online communities are digital collections of individuals that simultaneously satisfy the following four common characteristics, namely, the Internet as the material basis and the main activity place; information exchange is the link that maintains the online community; members of the online community have a sense of identity due to common needs; and members of the online community interact according to specific rules and methods to generate their own online community culture. From Tianya community, Douban, Tieba, various forums, BBS, and other online communities, to now based on WeChat, QQ, and a series of places that can attract people to gather, online communities have been formed, as shown in Figure 2.

Domestic and foreign studies have shown that online communities have educational functions, creating a platform for members in the group to learn interactively and generate collective knowledge, and the learning behavior of members in the group also creates the premise for the dissemination of knowledge and information, and the emergence of knowledge dissemination, research on knowledge sharing mode, sharing behavior influence mechanism, social reading development, invisible knowledge acquisition, interactive learning knowledge innovation, etc [10]. The academic community generally believes that the dissemination of information in the online community is related to the learning behavior of members in the group, and the learning behavior is determined by the three elements of individual characteristics, behavioral characteristics, and cultural environment and their interaction [11]. In recent years, some studies have paid attention to the application of network community education function in the field of ideological and political education and believe that its concealment and targeted advantages can be used as a new carrier of ideological and political education in colleges and universities, and an ideological and political education model under the network community should be actively constructed [12].

The research-based learning based on the network environment is a creative learning method cultivated through years of educational exploration and practice at the turning stage of revolutionary changes in science and technology and is an important practical form of educational informatization. Innovation is the soul of the development of the times and the fundamental need of scientific research and social development [13]. The core of innovation lies in creation. Among the many elements of creativity, the core is creative thinking. Creative thinking refers to the thinking process of solving problems with novel and original methods, which is an advanced form of human thinking. It refers to the comprehensive embodiment of multiple ways of thinking that reorganize existing knowledge and experience, propose new plans or procedures, and create new thinking results. Through this kind of thinking, people reveal the essential characteristics and regularity of things and phenomena, thus making discoveries and producing unprecedented thinking results.

## 3. The Rise of Online Community and Its Characteristic Analysis

According to the 45th “Statistical Report on Internet Development in China” released by CNNIC (Figure 3), as of March 2020, the number of netizens in my country reached 903 million, with a total of 31.17 million new netizens throughout the year [14]. The Internet penetration rate was 64.5%, an increase of 3.3 percentage points from the end of 2019. This means that nearly half of China's 1.36 billion people are netizens [15]. The Internet has assembled groups of individuals who were originally like the sands of the Ganges. With the support of the Internet, people's access to information is wider, easier, and cheaper.

When people enter into interaction, online communities are formed. The communication of the people in the real world generates the real society, and the transplantation extends to the Internet. Through the rapid information dissemination and exchange, a virtual community is formed—the human network social group. For example, QQ, Weibo, WeChat, and other users are the distinctive representatives of the online community. It is not only included in the network, but also an extension of the real social group, with the following new features.

### 3.1. Convenient Communication

The characteristics of the network make the network community have a good openness and a high degree of information sharing, break the boundaries of regions, and have a wide range of communication. Taking the rapidly developing WeChat as an example, it is not only a simple way to spread news in the past, but every user can continue to share each other's news in the circle of friends. The communication platform is simple and easy to operate. It is good at short messages, and the simple form of communication is quickly transformed into a fast and efficient communication mode. With the continuous development of 3G, 4G networks, and WEB2.0 technology (as shown in Figure 4), no matter the enterprise or individual, as long as there is a medium (mobile phone, tablet computer, desktop computer, etc.), they can chat on WeChat indefinitely. The network community represented by WeChat has a low threshold, which is easy to absorb users, and the huge user group spreads the message more widely [16].

### 3.2. Scalability

The infinite extensibility of the online community does make sense nowadays. In this illustration of a simulated network cluster, there are no clear edges, but can expand infinitely from the inside out. At the same time, it does not have a specified directionality, and it is a continuous transformation of the 360-degree comprehensiveness and the outside world [17]. Network data shows multidimensional correlations in both measurement and judgment and will spontaneously form connected small blocks that are separated from each other during the evolution process. This is of great significance for studying more social network models and understanding network collapse failure. “At the same time, semantics are formed by intermerging and connecting semantics from a large number of spontaneous individuals without global control and predefined madness, and the whole process continues to evolve as the data changes.” Every evolution of QQ, Weibo, WeChat, Twitter, and Facebook, social networking products at home and abroad, aims to make the service more suitable for ordinary users [18]. As the threshold continues to decrease, the number of user groups will continue to expand, as shown in Table 1.

### 3.3. Decentralization

After the rise of Web2.0, the services provided by network service providers such as Wikipedia, Flickr, and Blogger are all decentralized. Any participant can submit content, and netizens can jointly create or contribute to the content. Social media represented by QQ, Weibo, and WeChat have typical decentralization characteristics. Client users are both disseminators and audiences [19]. As a result, many people interact, presenting a complex honeycomb network structure, while scattered, diverse, and free subjects form the open, multifaceted, and borderless advantages of the network community. “In the online community, people can communicate many-to-many and realize multiperson interaction. The main body of communication also changes from real to virtual, from certain to unstable, from single to multiple, from centralized to decentralized.” Every client is a center that accepts and guides other clients around it; just like the mighty galaxy in the sky, it is pulled by a force in the dark. Everyone can participate, everyone can express, and everyone is an information provider, making the Internet structure more flat and challenging the traditional top-down community structure [20].

### 3.4. Difficult to Control

In the virtual space, netizens form various groups, circles, and interact in real time. However, the virtual space is not a face-to-face communication between people. For a social person, because there is no pressure from an actual identity, it is easier for people to expose their most real thoughts, and the Internet has become the best way to vent and express because everyone can speak and no one has verified the authenticity of the speech. This leads to uncontrollable news sources. The speed at which the Internet spreads makes the eventual reach of news uncontrollable. “The online community provides convenience for the information sharing of netizens and also allows some regional, local, and even accidental news events to spread rapidly through the online community, and the scope of influence continues to expand, forming “Internet hotspots” and attracting the attention of the whole people topic of public opinion”.

### 3.5. Self-Organization

German physicist Hermann Haken proposed the concept of synergy in 1971. He believes that if a system does not have external instructions, all parts of the system coordinate automatically according to certain rules and perform their duties to form an orderly structure, which is self-organization. Its formation process, driven by the internal mechanism, spontaneously changes from simple to complex, from disorder to order, and from low level to high level.

The network community as a whole reflects this characteristic. The process of forming from individual opinions to the formation of public opinion orientations shows the self-organization characteristics hidden in the network environment everywhere. The network community shows a strong self-organization and orderly self-organization.

## 4. Cultivation of Students' Innovative Thinking in the Online Community Environment

In work and life, innovative thinking is very important, it can solve the problems that plague us, that is, look at them in a different way or out of the way. There are seven innovative ways of thinking (as shown in Figure 5), each of which has its own characteristics and value, and can be mastered through learning and practice. Once learned and used, it will make your work and life easier and more comfortable and wonderful.

### 4.1. Use the Multidimensionality of the Network to Cultivate Students' Image Thinking, Intuitive Thinking, and Abstract Thinking

Image thinking is a way of thinking in which the human brain analyzes the appearance of objective things and then processes them into concrete images to solve problems. The way of image thinking to solve problems is imaginative activities. When solving problems, especially more complex problems, vivid and vivid images or representations are helpful for the smooth progress of the thinking process. Image thinking is mainly manifested in creative imagination and plays a very important role in artistic creation and technological innovation. Students should learn to use image thinking to solve their own scientific knowledge and practical problems in this subject, as shown in Table 2.

Intuitive thinking refers to the thinking activities of imagining, associating, comprehending, and judging new problems, new things, and new phenomena that appear in the process of problem exploration; the human brain often does not go through conscious and conscious logical reasoning. The use of intuitive thinking to quickly react and predict is not mysterious. It is a kind of direct comprehension and insight of the scientific research object by the conscious human brain. It reflects fast, accurate, agile, direct, and concise nature and suddenness. Because many intermediate links are omitted when solving problems, the basis is due to the individual's rich experience and profound scientific knowledge.

Abstract thinking, also known as theoretical thinking, abstract logical thinking, etc., refers to the thinking that uses concepts, judgments, and reasoning as the basic forms of thinking. Abstract thinking is unique to human beings and is the typical form of human thinking and the highest stage of individual thinking development. Students should develop the habit of observing and analyzing things, not only seeing the opposition and unity between things, as well as the positive and negative aspects of things, but also realizing the objective law that different things can be transformed into each other under certain conditions.

Research-based learning in the online community environment provides a platform for teachers and students to communicate, discuss, debate, and explore, promote students' research and exploration of problems more comprehensively and thoroughly, and can better cultivate students' innovative spirit and adapt to the demand for talents in the information age. It emphasizes that students make full use of virtual scientific experiments on the Internet to think and explore, so that they can generate intuitive thinking, image thinking, and abstract thinking through personal experience of learning activities.

### 4.2. Use the Multidimensionality of the Network to Expand the Thinking Space and Cultivate Students' Divergent Thinking

Innovative thinking is mainly based on divergent thinking, and the main characteristics of divergent thinking are seeking differences and innovation. Divergent thinking has no certain direction and scope, does not stick to conventions, and does not stick to traditional methods. It is a thinking that explores the unknown from the known. The evaluation of divergent thinking ability can be carried out from the three characteristics of thinking fluency, flexibility, and uniqueness. The fluency of thinking refers to thinking about many possible ideas per unit time, the number of ideas generated and the number of divergent items, and the utilization of stored data in the brain through insights and associations of things. Those who are fluent in thinking can move quickly, with smooth flow and less resistance, and can radiate more projects in a short period of time. Flexibility of thinking refers to “the ability of different categories or different ways of thinking to switch from one thought to another.” It refers to the scope or dimension of a project that diverges from a rigid way of thinking about problems and solutions. To solve problems, use flexible thinking methods to apply data and information, quickly adapt to various changing situations, and make different reflections and treatments for different problems. Those with flexible thinking are flexible and changeable by analogy in activities and are not bound by functional fixation. The uniqueness of thinking refers to imagining ideas that are unimaginable to others, and the divergent projects are beyond ordinary insights, with novelty, uniqueness, and high originality that are not similar to others. Only those who can be fluent can be flexible, and those who are both fluent and flexible can have extraordinary and unique insights.

### 4.3. Use the Multidimensionality of the Network to Cultivate Students' Original Thinking Personality and Critical Thinking Ability

Innovative thinking is the source of wisdom for all human inventions and creative activities, as shown in Table 3. Students use the Internet for research-based learning, which is conducive to broadening their knowledge horizons, getting rid of the confinement of book knowledge, breaking conventional thinking, and opening up their ideas and imagination. The Internet provides college teachers and students with a large amount of subject knowledge and rich academic resources, mobilizing students' enthusiasm and initiative in learning. Teachers should cultivate students' scientific attitude and literacy of seeking truth and pragmatism, which is of great significance to improving students' practical ability, innovation ability, and entrepreneurial ability.

First of all, cultivate students' original thinking personality. The highest state of innovative thinking is to cultivate students' originality, which is the inner foundation and essential characteristic of innovative thinking. Ingenuity refers to “thinking that goes beyond fixed, habitual patterns of cognition to ingeniously generate new, extraordinary thinking capabilities.” It manifests itself in generating novel, rare, and first-of-its-kind ideas and achievements. The deep-level network interaction environment can cultivate students' independent personality. Students communicate in an equal, free, and harmonious environment, and it is easy to form self-esteem and self-improvement personalities. It cultivates students to establish self-confidence and courage in the face of difficulties, and dare to accept difficulties and meet them. Challenge, stand up to your point of view and not submit to authority. The method of cultivating students' original thinking is to give full play to the students' spatial imagination ability, let the imagination plug in the wings of free flight, let the thinking run freely, and carry out independent creation. According to the teaching content and teaching progress, the students will be assigned homework related to their own creation, and the students will be guided to use the knowledge and skills they have learned to create original works independently, and the process of students' independent creation is the process of original thinking. Research-based learning is not only the transformation of learning methods and the cultivation of students' intelligence. Teachers must have a fraternal mind for students, be people-oriented, respect each student's unique personality, fully tap students' potential, and expand space for students' personality development.

Second, improve students' critical thinking ability. Critical thinking ability refers to “the thinking ability to evaluate conclusions by systematically and logically examining problems, evidence, and solutions.” If students lack critical thinking ability, it is impossible to ask more questions worthy of research, creating a research-oriented opportunity to learn. If the emphasis on judgment and reflection does not highlight innovation, it is not true judgment; on the contrary, if there is no judgment and reflection on existing outdated old concepts, there will be no innovation in thinking methods and thinking results. Intertwined with the outcomes of creative thinking, identifying problems and probing deviations in reasoning are key components of critical thinking.

In a word, to cultivate students' excellent intelligence and extraordinary talents, we must face all students, especially the underachievers, be people-oriented, respect people's nature and unique personality, explore people's creative potential, and create space for the full and free development of personality. Teachers should stimulate students' interest in exploration and cultivate innovative consciousness and the ability of image thinking, intuitive thinking, abstract thinking, divergent thinking, and critical thinking; through the training of forward thinking, reverse thinking, and multidirectional thinking, cultivate cooperation with others and form an initiative personality; encourage students to be innovative in academic issues, cultivate good at discovering and solving problems, dare to create a historical precedent, take the road that no one has gone before, and improve scientific literacy; cultivate a realistic and pragmatic scientific attitude and innovation ability and practical ability. However, if teachers lack the awareness of innovative thinking, it is impossible and unrealistic for students to form innovative thinking. Traditional education is often based on fractions, while research-based learning is the key for students to master active learning and explore a vast unknown space. Innovative thinking skills should be concerned by more and more people.

## 5. Conclusion

For China in the new era, it is dealing with the new contradiction between the people's ever-growing needs for a better life and unbalanced and inadequate development and undertakes important missions such as talent training, scientific research, social services, and cultural inheritance and innovation. Gathering young college students and intellectuals, it is at the forefront of the development of the technological revolution, the front line of the collision of Chinese and foreign cultures and the ideological struggle. In the era of big data, the online community has been deeply integrated with the thinking, study, work, and daily life of young college students. Making good use of the online community to cultivate innovative thinking is an important direction and key to the ideological and political education work in colleges and universities in the new era. The path is the practical need to implement the socialist core values. To this end, we must not only actively respond to the severe challenges brought by the “community” of online life, but also give full play to the ability and wisdom to use the online community for me. Find an entry point that meets the development needs of the new era in terms of organizational structure, topic construction, core character training, and the maintenance method of development centripetal force, and make good use of the online community as a carrier for the dissemination of socialist core values to give full play to the radiation effect.

## Figures and Tables

**Figure 1:** Analysis of the development environment of Chinese online communities.

**Figure 2:** Chinese online community industry members.

**Figure 3:** Scale of Internet users and Internet penetration rate.

**Figure 4:** The development history of social media.

**Figure 5:** Classification of innovative thinking.

**Table 1:** Comparison of social characteristics among Weibo, WeChat, and QQ.

Product name	Weibo	WeChat	QQ

Same	1. Support publishing content in plain text/graphics 2. You can beautify and edit pictures 3. Positioning information can be set 4. You can remind friends to check 5. You can set the visible range		

Different	1. The functional entrance is shallow, and it is the most conspicuous position on the APP homepage 2. Various image formats supported 3. Only 9 pictures can be posted, and the text limit is 2000 words 4. Cannot sync to other channels 5. It cannot be regularly published or deleted 6. Cannot add status labels 7. All Weibo users have the opportunity to view the posted messages 8. After setting to private state, it cannot be converted to public release, but the content set to public release can be converted to private state 9. The built-in function bar is rich in functions and supports adding articles, music, topics, etc. 10. In addition to the basic image beautification operations, there are various forms such as adding tags and links, and the options for image beautification are more abundant than the other two products.	1. The function entrance is deep, and the pure text publishing function entrance is hidden the deepest, which is the Easter egg function of WeChat to publish the circle of friends 2. Only support static image format 3. Only 9 pictures can be posted, and the text limit is 2000 words 4. It can be synchronized to its own product QQ space 5. It cannot be regularly published or deleted 6. Cannot add status labels 7. Only WeChat friends can view 8. After setting the visible range and publishing, it can be adjusted for the visible range (only for mutual settings of private and public states 9. The function of the built-in function bar is simple, only adding expressions	1. The function entrance is deep and scattered 2. Support two forms of static and dynamic pictures 3. You can publish more than 9 (unlimited) pictures, and the text limit is 10,000 words 3. It can be synchronized to the WeChat Moments of its own products 4. It can be published or deleted regularly 5. You can add status labels 6. QQ friends and QQ users who can access their space have the opportunity to view 7. After setting the visible range and publishing, it can be adjusted for the visible range |8. The built-in function bar is rich in functions and supports adding gif. voice talk, pattern fonts, etc.

**Table 2:** Evaluation indicators of online communities.

First-level indicator	Features/elements	Secondary indicators	Description	Reference source
Learning situation A	Teaching/teaching presence	Participation level A1	The performance of learners in daily speeches in online communities	Yu Shengquan. 2003; Jovanovic et al, 2012; Wei Shunping, 2015
		Complete homework A2	The learner is able to complete the coursework	
		Stage Test A3	The quality of learners completing stage tests	
Social event B	Sociability/social presence	Get appreciation B1	Learners can be appreciated by others	Yu Shengquan, 2003; Yiling, Xiaoqing, 2013
		Comment interaction B2	Learners interact with others	
		Content sharing B3	Learners share experiences, resources, etc., in the community	
Cognitive development C	Self-developmental/cognitive presence	Question C1	Learners are able to take the initiative to ask questions	Chen Wei, 2007; Lan Guoshuai, 2018
		Following the example C2	Learners imitate others to solve problems	
		Solve problem C3	Learners can spontaneously apply knowledge and skills to solve problems	

**Table 3:** Hierarchical framework of thinking quality.

Level	Types of thinking qualities	
Low level and high level	Observe	A perceptual activity of acquiring information is a purposeful, planned, and relatively lasting behavior.
	Compare	A method of judging the similarities and differences between two things.
	Analyze	A cognitive activity that divides the whole of the research object into various parts and examines them separately.
	Infer	The mental activity of reasoning and judging the causal relationship of facts based on facts or premises.
	Induction	Generalization of general concepts from individual things. A way of thinking about principles or conclusions.
	Concept construction	In the process of cognition, it rises from perceptual cognition to rational cognition, abstracts the common essential characteristics of perceived things, summarizes them, and forms an activity of conceptual thinking inertia.
	Critical thinking	A kind of reflective thinking that evaluates thinking according to certain criteria, and then improves thinking. With the existing thinking mode, using the existing knowledge and material, in a specific environment, propose something different from the conventional
	Innovative thinking	Or the opinions and methods of ordinary people.

## Data Availability

The labeled data set used to support the findings of this study is available from the corresponding author upon request.
